The article "Diagnostic Value and High-Risk Factors of Two-Dimensional Ultrasonography Combined with Four-Dimensional Ultrasonography in Prenatal Ultrasound Screening of Fetal Congenital Malformations" was published in 2022. Journal: Comput Math Methods Med.

# Diagnostic Value and High-Risk Factors of Two-Dimensional Ultrasonography Combined with Four-Dimensional Ultrasonography in Prenatal Ultrasound Screening of Fetal Congenital Malformations

**DOI:** 10.1155/2022/7082832

**Published:** 2022-07-12

**Authors:** Xinyou Yu, Fang Liu, Wei Gao, Xiangrong Shi, Ruiping Lu, Lihua Pan

**Affiliations:** ^1^Department of Prenatal Diagnosis Center, General Hospital of Ningxia Medical University, Yinchuan, 750004 Ningxia, China; ^2^Department of Reproductive Medicine, Yinchuan Maternity and Child Health Care Hospital, Yinchuan, 750004 Ningxia, China; ^3^Department of Ultrasound Examination, General Hospital of Ningxia Medical University, Yinchuan, 750004 Ningxia, China

## Abstract

**Objective:**

This study mainly analyzes the diagnostic value of two-dimensional ultrasonography (2D-US) combined with four-dimensional ultrasonography (4D-US) in prenatal ultrasound screening of fetal congenital malformations (CMs) and explores the high-risk factors affecting fetal malformations.

**Methods:**

The clinical and imaging data of 2247 pregnant women who underwent prenatal fetal malformation screening in the General Hospital of Ningxia Medical University between February 2020 and October 2021 were collected and analyzed, retrospectively. All pregnant women underwent 2D-US, and those with suspected fetal malformations were further inspected by 4D-US. The accuracy of ultrasound examination results relative to actual pregnancy outcomes was analyzed, taking the neonatal malformation after induced labor or actual delivery as the gold standard, and the risk factors influencing the occurrence of fetal malformations were discussed.

**Results:**

A total of 87 cases (3.87%) of fetal malformations were detected out of the 2247 parturients examined. The accuracy, sensitivity, and specificity of 2D-US diagnosis were 81.40%, 43.68%, and 82.92%, respectively, while the data were 83.67%, 51.72%, and 84.95% for 4D-US, respectively, and 93.59%, 90.80%, and 93.70%, respectively, for 2D-US +4D-US. The combined diagnosis of 2D-US +4D-US achieved statistically higher accuracy, sensitivity, and specificity than either of them alone. One-way analysis of variance and multivariate logistic regression analysis identified that the independent risk factors affecting fetal malformation were age ≥ 35, history of adverse pregnancy and childbirth, medication during pregnancy, toxic exposure during pregnancy, and history of seropositive for TORCH-IgM. Folic acid supplementation was a protective factor.

**Conclusions:**

Prenatal US is an effective approach for screening fetal malformations. 2D-US +4D-US can effectively improve the diagnostic rate of fetal malformations. For pregnant women with high-risk factors, prevention should be given priority, and prenatal screening and prenatal diagnosis should be standardized to reduce the occurrence of fetal malformations.

## 1. Introduction

Birth defects (BDs) are an important cause of infant mortality and lifelong disability [1]. According to the 2010 Global Burden of Disease Study, BDs, which lead to 6.4% of neonatal deaths, rank fifth among all causes of death [2] and place an enormous burden on families and society. Notably, the impact of BDs is particularly severe in low- and middle-income countries, including China. Approximately 900,000 babies are born with BDs every year in China, accounting for 5.6 percent of all births, according to a 2012 Report on The Prevention of Birth Defects in China [3]. Fetal structural malformation refers to fetal structural or chromosomal abnormalities occurring in utero due to its own genetic factors or maternal or external environmental factors, which accounts for over 90% of BDs and is one of the prime reasons for perinatal death. Studies have shown that about 2-3% of pregnancies are complicated with fetal structural abnormalities [4–6]. Generally speaking, it will lead to a series of deformities of different human systems in fetuses, such as nervous system, cardiovascular system, genitourinary system, and limb skeletal system, which has a great impact on the life and health quality of fetuses [7–9].

Ultrasound screening for fetal structural abnormalities is a routine component of prenatal care in resource-rich countries. Antenatal examination for structural abnormalities provides prospective parents with an opportunity to obtain early information about fetal structural abnormalities, including the nature, etiology, prognosis, and the feasibility of prenatal or postpartum treatment [10]. Prenatal screening can reduce the birth rate of malformed fetuses, which not only improves the quality of newborns but also promotes the development of every family and society at large [11]. Screening for chromosomal abnormalities is mainly based on the detection of serum in the second trimester of pregnancy. If abnormalities are indicated, further diagnosis can be made by amniocentesis or ultrasonography. Once the chromosome abnormalities is confirmed, the pregnancy will be terminated [12]. However, despite the high diagnostic accuracy of amniocentesis, puncturing or terminating a pregnancy in the second trimester can cause great harm to pregnant women, so finding a noninvasive and high-accuracy method for chromosomal abnormality screening is of utmost importance. As the most commonly used prenatal noninvasive examination method, ultrasound plays a critical role in fetal malformation and chromosome screening [13, 14]. At present, two-dimensional ultrasonography (2D-US) has become the main and routine method for prenatal screening because of its advantages of low cost, noninvasiveness and no X-ray exposure [15]. However, 2D-US is limited by the fact that its plane image can only show one side of the fetus, with limited detection metrics [16]. Studies have shown that the missed diagnosis or misdiagnosis of fetal craniocerebral abnormalities may be due to artifacts caused by umbilical cord interference [17]. Therefore, if fetal abnormalities are suspected on 2D-US and clearer images are needed for further evaluation, an examination modality with more advanced imaging capabilities is required. Four-dimensional ultrasonography (4D-US) is generated from continuous 3D images [18], which allows continuous monitoring of the fetal face and surface, including real-time movement and sharper images, giving a clear view of the fetus' overall appearance and fine structure [19]. 4D-US provides additional benefits in evaluating fetal prenatal condition [20]. However, the final performance of obstetric ultrasound images depends on various factors such as fetal recumbent position, uterine wall, abdominal wall fat, amniotic fluid, and number of gestational fetuses [21].

Therefore, if abnormalities are suspected on 2D ultrasound and clearer images and further evaluation are required, 4D ultrasound can be added to prenatal screening. This study retrospectively analyzed the ultrasonic features of 2247 pregnant women who were screened for prenatal fetal malformations. The main purpose was to explore the diagnostic effects of 2D-US and 4D-US on prenatal fetal malformations, and to compare the accuracy of their combined diagnosis and single diagnosis. Besides, we analyzed the risk factors related to malformations of fetuses with abnormal development, which is of great significance to improve the quality of birth population. The report is as follows.

## 2. Data and Methods

### 2.1. Study Population

The clinical and imaging examination data of 2247 pregnant women who underwent prenatal fetal malformation screening in the General Hospital of Ningxia Medical University between February 2020 and October 2021 were retrospectively analyzed. The age of the enrolled pregnant women was 20-40 years old, with an average of 30.09 ± 4.44 years old, and the gestational weeks ranged from 18 to 32 weeks, with a mean of 26.54 ± 2.13 weeks. In terms of the types of parturients, there were 1157 primiparas and 1090 multiparas. Inclusion criteria: (1) normal intrauterine pregnancy; (2) single pregnancy; (3) those who underwent 2D-US and 4D-US examinations; (4) complete clinical, imaging, and follow-up data. Exclusion criteria: (1) twin or multiple pregnancies; (2) severe heart, liver, and kidney diseases; (3) severe mental illness; (4) blood diseases and autoimmune diseases; (5) incomplete clinical, imaging, and follow-up data. This study was reviewed and approved by the hospital ethics committee.

### 2.2. Inspection Methods

A total of 2247 pregnant women were examined by Voluson E8 color Doppler ultrasound scanner (GE Healthcare, USA) with a probe frequency of 5.0-7.0 MHz. During the 2D-US examination, all patients were placed in the supine position with the abdomen exposed, and all aspects of the fetus were comprehensively scanned according to a common operation standard to carefully observe the state, structure, and size of each part of the fetus. The biological indicators of the fetus, such as biparietal diameter, head circumference, femur length, humerus length, abdominal circumference, placental position, and amniotic fluid index and maximum depth, were measured. The integrity of fetal skull was observed, and the ossification degree of fetal brain structure was detected. In addition, the head circumference, biparietal diameter, and posterior fossa depth were measured, the fetal face was observed in multiple sections, and the spine was checked for continuity. The normal development of chest structures such as heart and lungs, as well as the growth and development of the fetus were strictly evaluated. For pregnant women with suspected fetal malformations, 4D-US examination was carried out using a special probe RAB4-8-D with a frequency of 2.5-7.0 MHz. The dynamic imaging of the fetus was presented to ensure the clarity of the image acquisition. The accuracy of inspection results relative to induced labor and fetal indicators after delivery was compared and analyzed. All prenatal ultrasound examiners have received unified provincial training on prenatal ultrasound diagnosis. To ensure the accuracy of diagnosis, all cases were diagnosed by sonographers with provincial prenatal screening and diagnosis qualifications.

### 2.3. Endpoints

Pregnant women with possible fetal malformations indicated by prenatal B-ultrasound screening were followed up, and the accuracy, sensitivity, and specificity of 2D-/4D-US as well as their combined examinations in the diagnosis of fetal malformations were determined, with the neonatal malformation of pregnant women after induced labor or actual delivery as the gold standard. Accuracy = [(true positives + true negatives)/total cases] × 100%. Sensitivity = [true positives/(true positives + false negatives)] × 100%. Specificity = [true negatives/(true negatives + false positives)] × 100%.

The case data of pregnant women, including age, history of adverse pregnancy and childbirth, history of cold during pregnancy, history of medication during pregnancy, history of toxic exposure during pregnancy, and TORCH (toxoplasmosis, rubella, cytomegalovirus, and Herpes simplex virus) testing results of pregnant women, were investigated and analyzed by univariate and logistic regression analyses.

### 2.4. Statistical Analysis

The data of this study were tested by SPSS20.0 (IBM, NY, USA). Mean ± SD was used to represent measurement data; for count data recorded as *n* (%), the chi-square test was used for comparison. The threshold of significance was *P* < 0.05.

## 3. Results

### 3.1. Pregnancy Outcomes and Distribution of Fetal Malformations in Pregnant Women

A total of 87 cases (3.87%) of fetal malformations were detected in 2247 puerperae, including 21 neurological malformations, 15 cardiovascular malformations, 17 facial deformities, 5 digestive system malformations, 9 skeletal system deformity of extremities, 14 genitourinary system malformations, and 6 multiple malformations (Table 1). 2D-US imaging features of two malformed fetuses are shown in Figure 1.

### 3.2. Comparison of 2D- and 4D-US Diagnosis of Fetal Malformations

The comparison results between different inspection methods and the gold standard, namely, the occurrence of neonatal malformations after induced labor or actual delivery, were shown in Table 2. By calculation, it was found that the accuracy, sensitivity, and specificity of 2D-US diagnosis were 81.40%, 43.68%, and 82.92%, respectively, while the data for 4D-US were 83.67%, 51.72%, and 84.95%, respectively, and were 93.59%, 90.80%, and 93.70%, respectively, for 2D-US +4D-US. The combined diagnosis of 2D-US +4D-US achieved obviously higher accuracy, sensitivity, and specificity than either of them alone (Table 3).

### 3.3. Univariate Analysis of Risk Factors for Fetal Malformations

Univariate analysis showed that age ≥ 35, adverse pregnancy and childbirth history, folic acid (FA) supplementation, medication history during pregnancy, toxic exposure history during pregnancy, and history of seropositive for TORCH-IgM in pregnant women were related to fetal malformations, and the differences were statistically significant (*P* < 0.05), as shown in Table 4.

### 3.4. Multivariate Logistic Regression Analysis of Risk Factors for Fetal Malformations

Variables with significant differences in the univariate analysis were selected for further multivariate logistic regression analysis. It showed that age ≥ 35, history of adverse pregnancy and childbirth, history of medication during pregnancy, history of toxic exposure during pregnancy, and history of seropositive for TORCH-IgM in pregnant women were independently associated with increased risks of fetal malformations, while FA supplementation was a protective factor (*P* < 0.05), as shown in Table 5.

## 4. Discussion

Prenatal invasive diagnosis such as amniocentesis remains the gold standard for diagnosing fetal chromosomal abnormalities. However, amniocentesis is a traumatic procedure that carries a high risk of infection and abortion, so most pregnant women are reluctant to undergo it [22]. At present, 2D-US is a routine approach to screen fetal malformations before delivery. However, it can only provide a cross-sectional image of a certain part of the fetus, which cannot show the subtle structural features of the fetus, nor can it provide clearer and more effective stereoscopic images [23]. With the advancement of modern medical technology and the trend of refinement of medical devices, 4D-US has become an important supplement to 2D-US [24].

In this paper, 87 fetal malformations were detected among the 2247 parturients examined, accounting for 3.87%. The accuracy, sensitivity, and specificity of 2D-US diagnosis were 81.40%, 43.68%, and 82.92%, respectively, while were 83.67%, 51.72%, and 84.95%, respectively, for 4D-US, and 93.59%, 90.80%, and 93.70%, respectively, for 2D-US +4D-US. It indicates that the combined diagnosis of 2D-US +4D-US has significantly superior higher accuracy, sensitivity, and specificity to either 2D-US or 4D-US. These findings are consistent with those of Wang et al., who found that 2D-UD plus 4D-US can better identify various fetal brain abnormalities and provide early and more accurate information for clinicians and maternal patients to make decisions. In addition, 2D-US +4D-US has efficient application value in prenatal screening of fetuses at different gestational weeks. Deng et al. [25] found inferior diagnostic accuracy of 2D-US to 2D-US plus 4D-US for fetal anomaly at gestational week. Tudorache et al. [26] also reported that 2D-US and 4D-US are highly accurate tools for the early diagnosis of major congenital heart diseases by using high-quality systems and standard protocols.

This study also explored and analyzed the risk factors leading to fetal malformations. The results showed that age ≥ 35, adverse pregnancy and childbirth history, medication history during pregnancy, toxic exposure history during pregnancy, and history of seropositive for TORCH-IgM in pregnant women were all independent risk factors for fetal malformations, while FA supplementation was a protective factor. According to the study of Ge et al. [27], advanced pregnancy is a high-risk pregnancy that is more prone to neonatal developmental malformations. In most cases, environmental factors such as exposure to certain drugs, infections, or radiation during pregnancy can cause fetal deformities, though sometimes genetic [28]. The history of medication during pregnancy is also critical to the development of fetal malformations. Misuse of progesterones, estrogens, and androgens early in pregnancy may potentially lead to fetal brain and skull malformations [29]. However, it is inevitable for pregnant women with underlying diseases to take drugs to stabilize their condition. A study evaluating fetal malformations and seizure control in epileptic patients after discontinuation of sodium valproate (VPA) found that reducing the dose of VPA before pregnancy reduces the risk of fetal malformations, while discontinuation of VPA reduces harm to the general population, but at the cost of reduced seizure control during pregnancy [30]. This study also suggests that preventive measures should be taken when taking medicine during pregnancy, preferably by seeking medical advice. Multiple scientific evidence suggests that the environment may be associated with the occurrence of congenital malformations (CMs) such as limb deformities, orofacial clefts, and male genitourinary development, as well as with spontaneous abortion, which is more severe when parents are exposed to toxic pesticides [30, 31]. Parental exposure to toxic agrochemicals may increase the chances of children being born with CMs, particularly those related to the male reproductive system [32]. Maternal infections transmitted in utero by multiple pathogens at different stages of pregnancy are primarily responsible for newborn and infant deaths worldwide, with TORCH infections long associated with poor obstetric outcomes [33]. A prospective study on the relationship between TORCH infections and CMs in China demonstrated that TORCH infections are an important risk factor for severe fetal injury, especially CMs [34].

However, this study still has some limitations. First, we only studied patients during the second trimester of pregnancy and did not stratify the diagnostic value of 2D-US and 4D-US screening at different gestational weeks. Second, there were other risk factors that were not considered, such as radiation, smoking or drinking history of the husband, and genetic diseases. Thus, more research should be conducted to comprehensively analyze the diagnostic value of 2D-US and 4D-US in the screening of fetal congenital malformations.

## 5. Conclusion

To sum up, the combination of 2D- and 4D-DS can effectively improve the diagnosis rate of fetal malformations. The popularization of prenatal screening and timely prenatal diagnosis contributes to the reduction of newborn BDs. At the same time, pregnant women should stay away from environmental teratogenic factors and avoid all kinds of high-risk factors leading to fetal malformations and strengthen the awareness of prenatal and postnatal care, to improve the quality of birth population.

## Figures and Tables

**Figure 1:** Two-dimensional ultrasonic imaging features of malformed fetuses ((a) two-dimensional ultrasonography shows a “crab pincer” splitting of one foot; (b) two-dimensional ultrasonography shows severe dilation to the stomach and duodenum near the obstruction, with fluid retention and double bubble signs).

**Table 1:** Distribution of fetal malformations.

Classification of fetal malformations	Number of cases (*n*)	Constituent ratio (%)
Neurological malformation	21	24.14
Cardiovascular system malformation	15	17.24
Facial deformity	17	19.54
Digestive system malformation	5	5.75
Skeletal system deformity of extremities	9	10.34
Genitourinary system malformation	14	16.09
Multiple malformations	6	6.90
Total	87	100.00

**Table 2:** Comparison of 2D-US, 4D-US, and their combined detection results with pregnancy outcomes.

Examination method		Pregnancy outcomes		Total
		Positive	Negative	
2D-US	Positive	38 (1.69)	369 (16.42)	407 (18.11)
	Negative	49 (2.18)	1791 (79.71)	1840 (81.89)
4D-US	Positive	45 (2.00)	325 (14.46)	370 (16.47)
	Negative	42 (1.87)	1835 (81.66)	1877 (83.53)
Joint examination	Positive	79 (3.52)	136 (6.05)	215 (9.57)
	Negative	8 (0.36)	2024 (90.08)	2032 (90.43)

**Table 3:** Diagnostic efficacy analysis of different detection methods.

Examination method	Accuracy (%)	Sensitivity (%)	Specificity (%)
2D-US	81.40^∗^	43.68^∗^	82.92^∗^
4D-US	83.67^∗^	51.72^∗^	84.95^∗^
Joint examination	93.59	90.80	93.70

Note: ^∗^*P* < 0.05 vs. combination group.

**Table 4:** Univariate analysis of risk factors for fetal malformation.

Risk factors	Normal fetal group (*n* = 2160)	Malformed fetus group (*n* = 87)	*χ* ^2^	*P*
Age			22.7510	0.0069
<35	1651 (76.44)	47 (54.02)		
≥35	509 (23.56)	40 (45.98)		
Adverse pregnancy and childbirth history			29.3710	<0.0001
With	590 (27.31)	44 (50.57)		
None	1570 (72.69)	43 (49.43)		
Folic acid supplementation			7.9151	0.0049
Yes	705 (32.64)	41 (47.13)		
No	1455 (67.36)	46 (52.87)		
History of cold during pregnancy			1.9131	0.1666
Yes	882 (40.83)	42 (48.28)		
No	1278 (59.17)	45 (51.72)		
History of medication during pregnancy			54.9810	<0.0001
Yes	367 (16.99)	42 (48.28)		
No	1793 (83.01)	45 (51.72)		
History of toxic exposure during pregnancy			93.7010	<0.0001
Yes	77 (3.56)	22 (25.29)		
No	2083 (96.44)	65 (74.71)		
History			79.8510	<0.0001
Yes	74 (3.43)	20 (22.99)		
No	2086 (96.57)	67 (77.01)		

**Table 5:** Logistic regression analysis of risk factors for fetal malformations.

Risk factors	*β*	SE	*P*	OR	95% CI
Age (0: <35, 1: ≥35)	0.696	0.260	0.007	2.005	1.204-3.338
History of adverse pregnancy and childbirth (0: no, 1: yes)	2.076	0.637	0.001	7.974	2.288-27.793
Folic acid supplementation (0: no, 1: yes)	-3.232	0.790	0.000	0.039	0.008-0.186
Medication history during pregnancy (0: no, 1: yes)	2.117	0.530	0.000	8.306	2.941-23.461
Toxic exposure during pregnancy (0: no, 1: yes)	0.959	0.372	0.010	2.610	1.258-5.415
History of seropositive for TORCH-IgM (0: no, 1: yes)	0.831	0.348	0.017	2.296	1.160-4.542

## Data Availability

The labeled dataset used to support the findings of this study are available from the corresponding author upon request.

## References

[1] Mai C. T., Isenburg J. L., Canfield M. A. (2019). National population-based estimates for major birth defects, 2010–2014. *Birth Defects Research*.

[2] Lozano R., Naghavi M., Foreman K. (2012). Global and regional mortality from 235 causes of death for 20 age groups in 1990 and 2010: a systematic analysis for the global burden of disease study 2010. *The Lancet*.

[3] Yue W., Zhang E., Liu R. (2022). The China birth cohort study (cbcs). *European Journal of Epidemiology*.

[4] Rydberg C., Tunón K. (2017). Detection of fetal abnormalities by second-trimester ultrasound screening in a non-selected population. *Acta Obstetricia et Gynecologica Scandinavica*.

[5] Rayburn W. F., Jolley J. A., Simpson L. L. (2015). Advances in ultrasound imaging for congenital malformations during early gestation. *Birth Defects Research Part A: Clinical and Molecular Teratology*.

[6] Whitworth M., Bricker L., Mullan C. (2015). Ultrasound for fetal assessment in early pregnancy. *Cochrane Database of Systematic Reviews*.

[7] Cater S. W., Boyd B. K., Ghate S. V. (2020). Abnormalities of the fetal central nervous system: prenatal us diagnosis with postnatal correlation. *Radiographics*.

[8] Wang Y., Zhang J., Feng W. (2020). Description of misdiagnosis and missed diagnosis of fetal complex heart malformations by prenatal echocardiography combined with postnatal cardiovascular casting. *Prenatal Diagnosis*.

[9] Liu Y., Mapow B. (2020). Coexistence of urogenital malformations in a female fetus with de novo 15q24 microdeletion and a literature review. *Molecular Genetics & Genomic Medicine*.

[10] Edwards L., Hui L. (2018). First and second trimester screening for fetal structural anomalies. *Seminars in Fetal and Neonatal Medicine*.

[11] Cloutier M., Gallagher L., Goldsmith C., Akiki S., Barrowman N., Morrison S. (2017). Group genetic counseling: an alternate service delivery model in a high risk prenatal screening population. *Prenatal Diagnosis*.

[12] Zhang S., Yin M., Xu J.-Z. (2017). Cytogenetic analysis for fetal chromosomal abnormalities by amniocentesis: review of over 40,000 consecutive cases in a single center. *Reproductive and Developmental Medicine*.

[13] Drukker L., Bradburn E., Rodriguez G. B., Roberts N. W., Impey L., Papageorghiou A. T. (2021). How often do we identify fetal abnormalities during routine third-trimester ultrasound? A systematic review and meta-analysis. *BJOG: An International Journal of Obstetrics & Gynaecology*.

[14] Zhang N., Dong H., Wang P., Wang Z., Wang Y., Guo Z. (2020). The value of obstetric ultrasound in screening fetal nervous system malformation. *World Neurosurgery*.

[15] Vinals F., Ruiz P., Quiroz G. (2017). Two-dimensional ultrasound evaluation of the fetal cerebral aqueduct: improving the antenatal diagnosis and counseling of aqueductal stenosis. *Fetal Diagnosis and Therapy*.

[16] Sklar C., Yaskina M., Ross S., Naud K. (2017). Accuracy of prenatal ultrasound in detecting growth abnormalities in triplets: a retrospective cohort study. *Twin Research and Human Genetics*.

[17] Brandão P., Soares E., Estevinho C., Freixo M., Portela-Carvalho A. S., Ferreira M. J. (2018). Skeletal defect at mid-trimester ultrasound scan. *Journal of Medical Ultrasound*.

[18] Öcal D., Nas T., Güler İ. (2015). The place of four-dimensional ultrasound in evaluating fetal anomalies. *Irish Journal of Medical Science (1971-)*.

[19] Rossi A. C., Prefumo F. (2017). Correlation between fetal autopsy and prenatal diagnosis by ultrasound: a systematic review. *European Journal of Obstetrics & Gynecology and Reproductive Biology*.

[20] Vora N., Robinson S., Hardisty E., Stamilio D. (2017). Utility of ultrasound examination at 10-14 weeks prior to cell-free DNA screening for fetal aneuploidy. *Ultrasound in Obstetrics & Gynecology*.

[21] Bach-Ségura P. (2012). Facial clefts diagnosed before birth: routine ultrasound screening at the multi-disciplinary center for prenatal diagnosis (pcpd). *Journal of Dentofacial Anomalies and Orthodontics*.

[22] Rivas A., Epelman M., Danzer E., Adzick N. S., Victoria T. (2019). Prenatal mr imaging features of caroli syndrome in association with autosomal recessive polycystic kidney disease. *Radiology case reports*.

[23] Kurian J., Sotardi S., Liszewski M. C., Gomes W. A., Hoffman T., Taragin B. H. (2017). Three-dimensional ultrasound of the neonatal brain: technical approach and spectrum of disease. *Pediatric Radiology*.

[24] Barišić L. S., Stanojević M., Kurjak A., Porović S., Gaber G. (2017). Diagnosis of fetal syndromes by three-and four-dimensional ultrasound: is there any improvement?. *Journal of Perinatal Medicine*.

[25] Deng B., Hu D., Liu J., Lin H., Zhang Y., Li Z. (2015). Application of two-dimensional ultrasonography combined with four-dimensional ultrasonography in prenatal screening for fetal anomaly at different gestational weeks. *Evaluation and Analysis of Drug-Use in Hospitals of China*.

[26] Tudorache Ş., Cara M., Burada F., Simionescu C., Dragoescu A., Iliescu D. (2016). First trimester diagnostic accuracy of two-dimensional and four-dimensional ultrasound in major congenital heart diseases. *Obstetrics & Gynecology*.

[27] Ge G., Chen W., Jiang N. (2020). The value of prenatal color ultrasonography in the diagnosis of fetal structural malformation and the causes of missed diagnosis. *Acta Microscopica*.

[28] Tomà P., Bartoloni A., Salerno S. (2019). Protecting sensitive patient groups from imaging using ionizing radiation: effects during pregnancy, in fetal life and childhood. *La Radiologia Medica*.

[29] Yingjin W., Xiaoyuan C., Zhong R. Z. S., Yanyan P., Peili A., Xinru G. (2019). Diagnostic value of two-dimensional plus four-dimensional ultrasonography in fetal craniocerebral anomalies. *Iranian Journal of Public Health*.

[30] Ueker M. E., Silva V. M., Moi G. P., Pignati W. A., Mattos I. E., Silva A. M. C. (2016). Parenteral exposure to pesticides and occurrence of congenital malformations: hospital-based case–control study. *BMC Pediatrics*.

[31] Foster W. G., Evans J. A., Little J. (2017). Human exposure to environmental contaminants and congenital anomalies: a critical review. *Critical Reviews in Toxicology*.

[32] Costa N. Z., Nora C. R. D., Souto L. H. D., Carlotto F. D., Afonso R. . S., Riquinho D. L. (2021). Exposure to toxic agrochemicals and development of congenital malformations: a scoping review. *Texto & Contexto-Enfermagem*.

[33] Prasoona K. R., Srinadh B., Sunitha T. (2015). Seroprevalence and influence of torch infections in high risk pregnant women: a large study from South India. *The Journal of Obstetrics and Gynecology of India*.

[34] Wang Y., Li S., Ma N. (2019). The association of torch infection and congenital malformations: a prospective study in China. *European Journal of Obstetrics & Gynecology and Reproductive Biology*.

